# Service Sharing Decisions between Channels considering Bidirectional Free Riding Based on a Dual-Equilibrium Linkage Algorithm

**DOI:** 10.1155/2022/1540820

**Published:** 2022-06-27

**Authors:** Jing Zheng, Qi Xu

**Affiliations:** ^1^Glorious Sun School of Business and Management, Donghua University, Shanghai 200051, China; ^2^Logistics and E-Commerce College, Zhejiang Wanli University, Ningbo 315100, China

## Abstract

To solve the interchannel service-sharing decision problem, this paper constructs a dual-equilibrium linkage model between the static Stackelberg game and dynamic evolutionary game, considers the influence of bidirectional free riding and the proportion of service sharing the cost, and also studies the short-term equilibrium strategy and long-term stability strategy of the band owners and franchisees. The study indicates that, under the static Stackelberg model, as the cost of service sharing gradually decreases, the equilibrium strategy changes from the lose-lose situation of prisoner's dilemma to the Pareto Optimum of service sharing cooperation between the two parties. Under the dynamic evolutionary game, the offline free riding coefficient decreases, the cost-sharing ratio of the service sharing band increases, and the online free riding coefficient is still within the interval, and the stability result will change from the complete service competition to service sharing cooperation between channels.

## 1. Introduction

In recent years, global e-commerce has continued to grow at a high rate. According to the investigation report of Research (June 2019), the online retail sales in the Asia Pacific region will double in the next five years from $1.3 trillion in 2018 to $ 2.5 trillion in 2023, with a compound annual growth rate (CAGR) of 14.0%, accounting for 28% of the total retail sales. This has promoted more and more brand owners to redesign the structure of their traditional sales channels by participating in the online direct sales channels and to contact the customer groups that cannot be reached by traditional retail channels [1]. To cope with the threat of the brand owners' online channels, the retailers apply their offline channels to provide their consumers with additional services to help them better understand the product performance and promote the market sales [2]. Meanwhile, to be more attractive and competitive, different channels differ in their ability to perform various service outputs [3]. Therefore, when dual channels coexist, free riding is inevitable. The premise of free riding behavior is that the sales service provided by retailers can be separated from the final actual sales [4]. On the one hand, consumers collect relevant product information from online retailers and then buy such products online, which is also known as the showrooms effect [5]. For example, when consumers buy clothes, they may first go to physical stores to know the price of clothes and try them on and then turn to online channels with a lower price [6]. On the other hand, consumers obtain information services through the Internet but eventually buy offline, which is the result of the development of information technology that makes consumers more capable of obtaining information online, leading to free riding behavior of some consumers based on information services [7]. The practice has proved that 20.4% of offline sales occur due to the services provided by online channels, and 24.6% of online sales occur due to the services provided by offline channels [8], that is, the phenomenon of bidirectional free riding. Such bidirectional free riding intensifies competition among channels, which may further trigger horizontal competition between online direct sales channels and traditional retail channels, as well as vertical competition between manufacturers and retailers, and hinder supply chain members from acting as a whole system [9, 10]. However, little literature has focused on the bidirectional free riding in dual-channel supply chains.

To alleviate the service competition between channels, more and more brand owners have begun to explore the O2O model integrated with online and offline channels. By integrating online and offline channel resources, they can obtain the channel synergy advantages that cannot be met by a single channel, which can also meet the differentiated shopping needs of consumers and stimulate consumers' purchase behavior [11]. Therefore, in the O2O model, to encourage their offline franchisees to provide a showroom services, some brands share the service costs or provide service subsidies, such as INMAN, the famous Chinese Internet clothing brand, which shares part of the service costs of its offline franchisees (Sohu News) [12]. Meanwhile, in the O2O model, the brand owners would use the strong “flow effect” of online channels to encourage consumers to experience or buy in offline stores, while the offline retailer would provide the showrooms to eliminate the consumers' concerns about product quality when shopping online [13], realizing the integration of online and offline channel services and service sharing between the online and offline channels. However, when the online and offline channels belong to different subjects, that is, when the franchisee provides the showrooms as the brand's offline brick-and-mortar stores and also sells products as an independent retailer, the brand owner and the franchisee have both competitive and cooperative relationship, which will continue to remain. Then, from both short-term and long-term perspectives, can service sharing cooperation between channels be realized? And can the service cost sharing mechanism coordinate the conflict between the two parties?

In the existing research on dual-channel service sharing, the shared services are mainly offline channels providing showroom experience services for online channels and rarely consider online channels also providing drainage services for offline channels, resulting in the phenomenon of bidirectional free riding. The operation of dual channels is mainly based on retailers operating both online and offline channels at the same time and less considers the situation that online and offline channels are operated by different entities. The main research perspective is single perspective, such as static perspective (Nash equilibrium) or dynamic perspective (differential game or evolutionary game), and there are few studies from dual perspective and dual-equilibrium perspective. To fill these gaps, this paper considers a brand that sells its products through its online channel and offline franchised stores, and there is a bidirectional free rider situation between online and offline channels, and the brand and franchised stores present a complex competitive cooperation relationship. Considering the degree of bidirectional free riding, from both static and dynamic perspectives, brands and franchised stores make competing decisions on service sharing issues. Finally, whether the service cost sharing mechanism can achieve reconciliation of conflicts between the two parties and ultimately achieve Pareto optimality is discussed. This study contributes to the literature from four perspectives:

1. A dual channel consisting of brand owners and franchisees is constructed, and the complex competition between such dual channels with different subjects is investigated compared to dual channels with the same subject in terms of service sharing.
2. Complementing the study of bidirectional free ridership in dual-channel supply chains, we focus on the impact of the degree of free ridership on interchannel service sharing decisions.
3. From the perspective of the static game and dynamic game equilibrium, we analyze the competing relationship and the impact of decision-making of supply chain members in service sharing between channels, which is more comprehensive and feasible than the analysis from a single perspective.
4. A cost sharing mechanism to coordinate the competition and decision-making of supply chain members is proposed.

The structure of the remainder of the paper is as follows: Section 2 reviews the relevant literature. In Section 3, the research question is described in detail.  Section 4 analyzes the service sharing decision-making of brand owners and franchisees from the perspective of static equilibrium and discusses the impact of relevant parameters on them.  Section 5 is about dynamic evolutionary game analysis, analyzing the service sharing decision-making of brand owners and franchisees from the perspective of dynamic equilibrium, and discussing the impact of relevant parameters on them. Finally, Section 6 summarizes the research results and their practical significance and puts forward the direction of future research.

## 2. Literature Review

This study mainly involves three research areas: the free riding phenomenon, the O2O model, and the competition and cooperation relationship between dual channels. We briefly review the literature on these three aspects.

The free riding phenomenon in the supply chain was first proposed by Telser, who believes that this phenomenon was not conducive to the enthusiasm of retailers to provide information services. Through the retailer price maintenance agreement, the service quality is limited and not reduced [14]. At present, the main research object of free riding in the supply chain is the negative impact of free riding, which means that free riding behavior will damage the interests of service retailers [6, 15, 16]. Some scholars also proposed different views that free riding can alleviate the fierce price competition between retailers providing information services and free riding retailers. The above literature only studies the free riding phenomenon between traditional brick-and-mortar retailers [17, 18]. With the rapid development of e-commerce, scholars began to study the impact of dual-channel free riding on supply chain performance. For the channel conflict caused by it, the coordination mechanism is designed to weaken the free rider problem. Common coordination mechanisms such as cost sharing contracts [19–21] and the combination of repurchase contracts, sales rebates, and other contracts can optimize the retailer's effort level [22–24], while Wang and Gerchak used the supplier to compensate the retailer's effort cost through inventory subsidy [25]. The above literature research is a unidirectional free riding problem between dual channels, that is, the showrooms' effect on the decision-making of members of the dual-channel supply chain [26–28]. The revelation effect is a special way of free riding [29]. The bidirectional free riding problem is mainly the bidirectional free riding problem among retailers [8, 30]. While the problem of bidirectional free riding in dual channels is rarely studied, Bernstein et al. defined the bidirectional free riding behavior and they thought that when the product information services provided by the traditional retail channel and the online channel are complementary, the bidirectional free riding behavior based on information services between the channels is inevitable [31]. Liu et al. studied the pricing strategy of dual-channel supply chains considering fairness factors and free riding behavior when the manufacturer's direct sales network channel and traditional retail channel coexist [32]. The possibility of bidirectional free riding in Internet finance was studied by Yan et al. [33].

In the traditional dual-channel supply chain, consumers often enjoy experiential services in the offline channel and then turn to the online channel to make purchases. This free-riding behavior of consumers has intensified the competition between channels. Therefore, the O2O model has realized the integration of online and offline channel services or the service sharing from the online channel to the offline channel or from the offline channel to the online channel. At present, the O2O cooperation forms are mostly studied in the cooperation mode of “online purchase and offline pick-up” from online to offline and the cooperation mode of “online purchase and offline experience” from offline to online; among them, the existing online to offline research mainly focuses on the impact of O2O model on consumers' purchase behavior, channel demand, and decision-making of relevant stakeholders. For example, Gallion analyzed the impact of the cooperation mode of “online purchase and offline pick-up” on consumers' purchase behavior and retailers' demand in different channels [34]; Gao and Cao, respectively, studied the impact of the cooperation mode of “online purchase and offline pick-up” on retailers' optimal inventory decision-making and optimal pricing decision-making [35, 36]. The existing research from offline to online mainly focuses on the impact of O2O model on consumers' return behavior, inventory or pricing decision-making, and the design of incentive mechanisms in the process of O2O model cooperation. Bell et al. took Warby Parker as an example [37] and Chopra took Bonobos as an example [38] to study the impact of the cooperation mode of “offline experience and online purchase” on consumers' return behavior and enterprise operation efficiency. Gao and Su and Dan et al. studied the optimal inventory decision under the “offline experience, online purchase” model [39, 40]. For a retailer with both online and offline channels, Du and others have analyzed the impact of consumer disappointment and aversion caused by uncertain product value on the retailer's pricing strategy and discussed the role of introducing the cooperation mode of “offline experience and online purchase” [41]. Li et al. investigated the optimal pricing decision of a competitive supply chain between offline experience stores and online retailers [42]. However, these papers mainly focus on the channel cooperation when online and offline belong to the same subject, which is the O2O cooperation between online retailers and offline experience stores, while such experience stores do not directly sell the same products as online but only provide product experience for online products. In reality, some brand owners with online direct sales channels, such as INMAN and Blue Nile, sell the same products with the offline franchisees. Therefore, there is competition and cooperation between the channels, which is more complicated than the relationship between online retailers and specialized offline experience stores that only have cooperation.

Some scholars have considered the impact of product competition on O2O supply chain management in the “offline experience, online purchase” model. Dan et al. discussed whether online brand owners should cooperate with retailers selling competitive products to open experience stores [43]; Zhang et al. studied the response strategies of online brands when they cooperated with retailers to set up experience stores and retailers introduced competitive products [44]. Some scholars also considered the influence of competition among suppliers on O2O supply chain management under the mode of “offline experience and online purchase.” For example, Li et al. studied whether the offline experience stores with asymmetric information should introduce a new competitive online retailer to meet the differentiated needs of consumers [45]. Liu found in his study that free riding can promote the increase of total market demand, but it has a differentiation effect on the offline demand. To solve this contradiction, he proposed a cooperation strategy that can effectively eliminate the negative impact of free riding and enable both parties to achieve Pareto improvement [46].

Currently, the service sharing on dual channels mainly focuses on static short-term perspectives. For example, Long and Shi studied the cooperation conditions, pricing strategies, and benefits when tour operators (TOs) and online travel agencies (OTAs) realized O2O model through online sales and offline service cooperation by constructing Stackelberg and Bertrand competitive game models [47]. Kong et al. analyzed the optimal pricing and service decisions under centralization and decentralization for dual channels of closed-loop supply chains, respectively [48]. Vamvakas et al. used the noncooperative CPR game between users to solve the corresponding noncooperative game and prove that it converges into a unique pure Nash equilibrium point [49]. A dynamic long-term perspective is rarely studied. Ma et al. analyzed the performance of a supply chain system under the O2O framework based on Bellman's continuous dynamic programming theory for the manufacturer's quality strategy, the retailer's service level strategy, and the three decision models of decentralization, centralization, and reciprocal altruism [50].

To sum up, brands adopt the O2O model to complete online to offline drainage services. The offline franchisees complete the offline to online experience services by providing the showrooms. Both sides realize interchannel service sharing cooperation. However, due to the competitive and cooperative relationship between the brands and franchises, as well as the existence of bidirectional free riding, the competitive and cooperative game relationship between both parties is more complex. The goal is no longer static coordination but dynamic continuous optimization and coordination. Therefore, based on the literature review, this study considers the impact of bidirectional free riding on the service sharing decision in dual-channel supply chains from the static and dynamic perspectives.

## 3. Model Building

### 3.1. Problem Description

Suppose that a two-level supply chain system consists of a brand supplier and its offline stores. The brand supplier sells products through its online channel and offline stores. The offline stores studied in this paper are franchised, at which point there is a cooperative and competitive relationship between the brand owner and the offline franchised stores. The brand wholesales products to the franchisee at price *ω*, and the franchisee sells products to the consumers at price *P*_*r*_. The brand owner itself sells at price *P*_*d*_ in its online direct sales channel and satisfies *ω* ≤  *P*_*d*_ < *P*_*r*_. The brands' O2O (online to offline) model encourages online customers to experience or consume in offline stores and provides drainage services *S*_*d*_ for the offline channel. The franchisees provide offline exhibition hall services *S*_*r*_ to realize service sharing among online and offline channels. Service sharing emphasizes that service cooperation between channels is different from service competition or free riding between channels. The research focus on service sharing decisions in the dual-channel supply chain is shown in Figure 1 and the notations are summarized in Table 1.

The linear demand function is usually jointly determined by price and sales effort, and such a linear function of deterministic market demand is adopted [21, 48, 51]. Based on the above assumption, the linear demand function of the channel in this paper is jointly determined by price, service level, and the degree of service sharing between channels, described as follows:

(1) $$\begin{array}{c} Q_{i}=1-P_{i}+\beta P_{j}+\left(1-\lambda_{i}\right)S_{i}+\lambda_{j}S_{j},\left(i,j=d,r;i\neq j\right). \end{array}$$

In the above formula, *Q*_*i*_(*i*, *j*=*d*, *r*) are the demands of online and offline channels, respectively. *β*(0 < *β* < 1) denotes the price sensitivity coefficient between channels. The larger the *β* value is, the more intense the price competition between channels is. (1 − *λ*_*i*_) denotes the service effort coefficient of the channel. *λ*_*i*_(0 < *λ*_*i*_ < 1) denotes the free riding coefficient between channels.

When channel *i*(*i*=*d*, *r*) provides service *S*_*i*_, in addition to bringing its demand increase (1 − *λ*_*i*_)*S*_*i*_, channel *j* will also serve free riding to increase the demand of *λ*_*i*_*S*_*i*_. To simplify the analysis, it is assumed that service *S*_*i*_ obeys the two-point distribution. When the channel provides services, *S*_*i*_=*S*(*i*=*d*, *r*) and the service cost is *C*_1_. Otherwise  *S*_*i*_=0 and the service cost is 0.

In this paper, the brand and franchisee have a complex relationship of competition and cooperation and make decisions by weighing costs and benefits. To simplify the analysis without loss of generality, it is assumed that the marginal production cost of the brand and the marginal sales cost of the franchisees are 0 [40, 52]. When the brand owners and franchisees cooperate to realize the service sharing, the total cost of service sharing is set as *C*, which is shared by both parties [53]. The cost sharing ratio of the brand is *ξ*0 < *ξ* < 1, while the franchisee takes the ratio of (1 − *ξ*). We assume that (1 − *ξ*)*C* < *C*_1_ and  *ξC* < *C*_1_.

### 3.2. Model Building

According to the above problem description, this paper assumes that the brand is the dominant player in the supply chain and the franchisee is the follower. The brand decides whether to adopt the O2O model to realize online to offline drainage services, while the franchisee decides whether to provide showroom services to realize offline to online experience services. Therefore, the two decision-making bodies form four different strategies, which are specifically described as follows.

*G* ^*N*^ *H* ^*N*^ refers to the competition-competition relationship between brands and franchisees. That is, brands adopt a dual-channel model and franchisees do not provide showroom services. The profits of the brand and franchisee are given as follows:

(2) $$\begin{array}{c} \Pi_{M}=P_{d}Q_{d}+\omega Q_{r};\;\Pi_{R}=\left(P_{r}-\omega \right)Q_{r}. \end{array}$$

*G* ^*N*^ *H* ^*Y*^ indicates that the brand and franchisee are in a competition-cooperative relationship. That is, the brand adopts the dual-channel model, while the franchisee provides the showroom service. The profits of the brand and franchisee are given as follows:

(3) $$\begin{array}{c} \Pi_{M}=P_{d}Q_{d}+\omega Q_{r};\Pi_{R}=\left(P_{r}-\omega \right)Q_{r}-C_{1}. \end{array}$$

*G* ^*Y*^ *H* ^*N*^ indicates that the brand and franchisee are in a cooperative-competition relationship. That is, the brand adopts the O2O model, while the franchisee does not provide the showroom service. The profits of the brand and franchisee are given as follows:

(4) $$\begin{array}{c} \Pi_{M}=P_{d}Q_{d}+\omega Q_{r}-C_{1};\;\Pi_{R}=\left(P_{r}-\omega \right)Q_{r}. \end{array}$$

*G* ^*Y*^ *H* ^*Y*^ indicates that the brand and franchisee are in a cooperative-cooperative relationship. That is, the brand adopts the O2O model, while the franchisee provides the showroom service. The profits of the brand and franchisee are given as follows:

(5) $$\begin{array}{c} \Pi_{M}=P_{d}Q_{d}+\omega Q_{r}-\xi C;\Pi_{R}=\left(P_{r}-\omega \right)Q_{r}-\left(1-\xi \right)C. \end{array}$$

## 4. Static Equilibrium Strategy

This section analyzes how the brand and the franchisee price to maximize their profits under the four strategies. In this paper, the reverse induction method is used to solve the problem. As the leader of the Stackelberg game, the brand first determines the wholesale price *ω* and the online direct sales price *P*_*d*_. The franchisee determines the offline retail price *P*_*r*_ later.

**Proposition 1 .**

The optimal pricing under each strategy combination is shown in Table 2.

**Proof**

See Appendix A.

**Conclusion 1 .**

By comparing the optimal pricing under different strategy combinations of the brand and the franchisee, the following relationship can be obtained.

When the service effort coefficient (1 − *λ*_*i*_) or the free riding coefficient *λ*_*j*_ satisfies 1/2 < 1 − *λ*_*d*_ < *λ*_*r*_ < 1, the relationship between the wholesale price  *ω*, online direct selling price  *P*_*d*_, and offline retail price *P*_*r*_  of each strategy is as follows:

(6) $$\begin{array}{c} \omega^{YY*}>\omega^{YN*}>\omega^{NY*}>\omega^{NN*},\\ P_{d}^{YY*}>P_{d}^{NY*}>P_{d}^{YN*}>P_{d}^{NN*},\\ P_{r}^{YY*}>P_{r}^{YN*}>P_{r}^{NY*}>P_{r}^{NN*}. \end{array}$$

If the condition satisfies 1/2 < *λ*_*r*_ < 1 − *λ*_*d*_ < 1, the optimal price relationship of each strategy is obtained as follows:

(7) $$\begin{array}{c} \omega^{YY*}>\omega^{NY*}>\omega^{YN*}>\omega^{NN*},\\ P_{d}^{YY*}>P_{d}^{YN*}>P_{d}^{NY*}>P_{d}^{NN*},\\ P_{r}^{YY*}>P_{r}^{NY*}>P_{r}^{YN*}>P_{r}^{NN*}. \end{array}$$

**Proof**

See Appendix B.

This indicates that the optimal pricing of strategy *G*^*Y*^*H*^*Y*^ is the highest and strategy *G*^*N*^*H*^*N*^ has the lowest optimal pricing under different strategy combinations. The optimal pricing of strategy *G*^*Y*^*H*^*Y*^ and that of strategy *G*^*N*^*H*^*N*^ are affected by the service effort coefficient 1 − *λ*_*j*_ and the free riding coefficient *λ*_*i*_ between channels.

Both the brand and franchisee need to invest a lot of costs to realize service sharing between channels. To protect the profit margin, both parties will be priced at the highest level. Similarly, if neither the brand nor the franchisee provides shared services, both parties do not have to invest the relevant costs and both parties have the lowest pricing. However, the situation is more complex when the brand and franchisee are in a competitive and cooperative relationship. If the sharing service provided by the brand has less impact on the growth of online channel demand than the franchisee (i.e., 1 − *λ*_*d*_ < *λ*_*r*_), the brand is more willing to encourage the franchisee to provide shared services. The brand will give lower prices *ω* so that the franchisee can also reduce price *P*_*r*_. The brand adjusts price *P*_*d*_ to alleviate the price competition with the offline channel and make up for the profit loss caused by the reduction of the wholesale price. On the contrary, the brand prefers adopting the O2O model to provide shared services, which will offer higher price *ω* and reduce price *P*_*d*_ to enhance competitiveness with the offline channel. The franchisee has to raise price *P*_*r*_ due to the increase in the whole price.

**Proposition 2 .**

The optimal pricing under each strategy is shown in Table 3.

**Proof**

See Appendix A.

**Conclusion 2 .**

By comparing the optimal profit under different strategy combinations, the optimal strategy of the brand and the franchisee can be obtained:

1. Considering the optimal profit of the brand, Π_*M*_^*NN∗*^ < Π_*M*_^*NY∗*^ and Π_*M*_^*YN∗*^ < Π_*M*_^*YY∗*^ are established. Satisfying *C* > *E*_1_, the brand prefers strategy *G*^*N*^*H*^*Y*^, and satisfying *C* < *E*_1_, the brand prefers strategy *G*^*Y*^*H*^*Y*^.
2. Considering the optimal profit of the franchisees, Π_*R*_^*NN∗*^ < Π_*R*_^*YN∗*^ and Π_*R*_^*NY∗*^ < Π_*R*_^*YY∗*^ are established. Satisfying *C* > *E*_2_, the franchisee prefers strategy *G*^*Y*^*H*^*N*^, and satisfying *C* < *E*_2_, the franchisee prefers strategy *G*^*Y*^*H*^*Y*^.

In the above, *E*_1_=*S*(*S*(3 − 4*β*+*β*^2^)*λd*^2^ − 2(1 − *β*)*λd*((1+*S*)(1+*β*)+*S*(3 − *β*)*λr*)+2(2+*S*+2*β*+2*Sβ*+2*S*(1 − *β*)*λr*))/8(1 − *β*^2^)*ξ*. Ans *E*_2_=*S*(1 − *λ*_*r*_)(2+*S*+2*Sλ*_*d*_ − *Sλ*_*r*_)/16(1 − *ξ*).

**Proof**

See Appendix B.

It is shown that the optimal profit of the brand and the franchisee is affected by the total cost *C* of service sharing between channels. When the value of *C* is high, both the brand and the franchisee prefer providing shared services only to each other, namely, strategy *G*^*Y*^*H*^*N*^ or strategy *G*^*N*^*H*^*Y*^. With the in-depth cooperation between them, the total cost *c* of service sharing between channels gradually reduces, and they become more inclined to win-win cooperation, namely, strategy *G*^*Y*^*H*^*Y*^.

**Conclusion 3 .**

The equilibrium strategies of the brand and the franchisee are affected by the shared service cost *C* and the channel service cost *C*_1_, as shown in Figure 2. When *C* < *E*_2_, the system equilibrium strategy is *G*^*Y*^*H*^*Y*^. If *C* > *E*_2_ and *C*_1_ > *E*_3_, the system equilibrium strategy is *G*^*N*^*H*^*N*^. When *C* > *E*_2_ and *C*_1_ < *E*_3_, the system equilibrium strategy is *G*^*Y*^*H*^*N*^.

In the above, *E*_3_=*S*(2(2+*S*+2*β*) − 2(1 − *β*)(1+2*S*+*β*)*λ*_*d*_+*S*(3 − 4*β*+*β*^2^)*λ*_*d*_^2^)/8(1 − *β*^2^)  and *E*_4_=*S*(1 − *λr*)(2+*S* − *Sλ*_*r*_)/16, when *E*_4_ < *E*_3_.

**Proof**

See Appendix B.

According to Conclusions 2 and 3, the optimal strategy and the system equilibrium strategy are compared. When *C*(*C* > *E*_2_) is comparatively large, the prisoner's dilemma appears. At this point, the brand's optimal strategy, the franchisee's optimal strategy, and the system equilibrium strategy are inconsistent. With the deeper cooperation between the brand and franchisee, the service sharing cost C (*C* < *E*_2_) gradually decreases. At this point, the optimal strategy and system equilibrium strategy of both parties are *G*^*Y*^*H*^*Y*^ strategies to achieve the Pareto optimality.

**Conclusion 4 .**

With the decrease of the free riding coefficient *λ*_*d*_ of the offline channel, the final system equilibrium tends to be strategy *G*^*Y*^*H*^*N*^; that is, the brand adopts the O2O model, while the franchisee does not provide showroom services. However, if *λ*_*d*_ increases, the final system equilibrium tends to be strategy *G*^*Y*^*H*^*Y*^; that is, the brand adopts the O2O model and the franchisee provides showroom services.

**Conclusion 5 .**

With the decrease of the free riding coefficient *λ*_*r*_ of the online channel, the final system equilibrium tends to be strategy *G*^*Y*^*H*^*N*^; that is, the brand adopts the O2O model, while the franchisee does not provide showroom services. However, if *λ*_*r*_ increases, the final system equilibrium tends to be strategy *G*^*Y*^*H*^*N*^; that is, the brand adopts the O2O model and the franchisee provides showroom services.

**Proof**

See Appendix B.

According to Conclusions 4 and 5, the change of online and offline free riding coefficient makes the system equilibrium strategy inclined to dual-channel services sharing cooperation or provide shared services only through the online channel. This is mainly because the brand, as the supply chain leader, prefers adopting the O2O model to enhance the consumer experience, thereby driving growth in overall supply chain performance. As followers, whether the franchisee provides showroom services is affected by the degree of online and offline free riding. If there is a greater degree, the franchisee is more willing to cooperate with the brand and realize service sharing cooperation. In this case, the system equilibrium strategy tends to be strategy *G*^*Y*^*H*^*Y*^. Conversely, if the degree of free riding in offline channels is greater, the franchisee is more inclined not to provide showroom services. At this point, the system equilibrium strategy tends to be strategy *G*^*Y*^*H*^*N*^.

**Conclusion 6 .**

With the decrease of price sensitivity coefficient *β* between channels, the final system equilibrium strategy tends to be strategy *G*^*N*^*H*^*N*^; that is, the brand owner adopts dual-channel model, while the franchisee does not provide showroom services. However, if *β* increases, the final system equilibrium strategy tends to be strategy *G*^*Y*^*H*^*N*^; that is, the brand adopts the O2O model, while the franchisee does not provide showroom services.

Due to *P*_*d*_ < *P*_*r*_, *β* has no impact on the decision of the franchisee, and it always prefers not to provide showroom services. However, the change in price sensitivity coefficient between channels will have an impact on the decision of the brand. When *β* decreases, the price advantage of the brand has less and less impact on the growth of online demand, as well as the possibility of online free riding. At that time, brand owners prefer not to provide shared services, and the final system equilibrium strategy tends to be strategy *G*^*N*^*H*^*N*^. With the increase of price sensitivity coefficient *β* between channels, the possibility of online free riding increases; that is, the brand is more willing not to implement service sharing cooperation, and the final system equilibrium strategy tends to be strategy *G*^*Y*^*H*^*N*^.

**Conclusion 7 .**

With the proportion of service sharing cost *ξ* of the brand decreasing, the final system equilibrium strategy tends to be strategy *G*^*N*^*H*^*N*^; that is, the brand adopts the O2O model, while the franchisee does not provide showroom services. However, if *ξ* increases, the final system equilibrium strategy tends to be strategy *G*^*Y*^*H*^*Y*^; that is, the brand adopts the O2O model, while the franchisee provides showroom services.

For the long-term development of the brand, it prefers to implement service sharing cooperation. When *ξ* decreases, it means that the proportion of service sharing cost (1 − *ξ*) of the franchise increases. The franchisee gradually tends not to provide showroom services; that is, the system equilibrium strategy tends to be strategy *G*^*Y*^*H*^*N*^. When *ξ* increases, the franchisee's proportion (1 − *ξ*) decreases, making the franchisee willing to cooperate and provide showroom services; that is, the system equilibrium strategy tends to be strategy *G*^*Y*^*H*^*Y*^.

## 5. Dynamic Equilibrium Analyses

Under normal circumstances, game players have limited rationality and do not have enough information or the ability to make optimal decisions [54]. Therefore, the equilibrium strategy among game players cannot be obtained through a single game but through continuous learning and dynamic adjustment in multiple rounds of games. This section uses the cooperative evolutionary game to analyze the optimal decision of the brand and the franchisee.

### 5.1. Analysis of Evolutionary Game Strategy

Based on behavioral economics, this section assumes that the brand and the franchisee can make optimal decisions independently and repeat the game for continuous cooperation in the future. Specifically, it is assumed that the probabilities of the brand adopting “O2O model” and “dual-channel model” strategies are *x*(0 ≤ *x* ≤ 1) and 1 − *x*. Meanwhile, the probabilities of the franchisee adopting the strategies of “showroom service” and “no showroom service” are *y*(0 ≤ *y* ≤ 1)  and 1 − *y*. The adaptability of strategy is expressed by profit, and the payoff matrix is simplified as in Table 4.

The fitness of “O2O model” strategy is

(8) $$\begin{array}{c} E\left(G^{Y}\right)=y\Pi_{M}^{YY*}+\left(1-y\right)\Pi_{M}^{YN*}. \end{array}$$

The fitness of “dual-channel model” strategy is

(9) $$\begin{array}{c} E\left(G^{N}\right)=y\Pi_{M}^{NY*}+\left(1-y\right)\Pi_{M}^{NN*}. \end{array}$$

The average fitness is

(10) $$\begin{array}{c} E\left(G\right)=xE\left(G^{Y}\right)+\left(1-x\right)E\left(G^{N}\right). \end{array}$$

The fitness of “showroom Service” strategy is

(11) $$\begin{array}{c} \;E\left(H^{Y}\right)=x\Pi_{R}^{YY*}+\left(1-x\right)\Pi_{R}^{NY*}. \end{array}$$

The fitness of “no showroom Service” strategy is

(12) $$\begin{array}{c} E\left(H^{N}\right)=x\Pi_{R}^{YN*}+\left(1-x\right)\Pi_{R}^{NN*}. \end{array}$$

The average fitness is

(13) $$\begin{array}{c} E\left(H\right)=yE\left(H^{Y}\right)+\left(1-y\right)E\left(H^{N}\right). \end{array}$$

Therefore, the repeated dynamic differential equation of the brand and the franchisee is as follows:

(14) $$\begin{array}{c} F_{1}\left(x,y\right)=\frac{\text{d}x}{\text{d}t}=x\left(1-x\right)\left[y\left(\Pi_{M}^{YY}-\Pi_{M}^{NY}\right)+\left(1-y\right)\left(\Pi_{M}^{YN}-\Pi_{M}^{NN}\right)\right],\\ F_{1}\left(x,y\right)=x\left(1-x\right)\left[P_{d}S\left(1-\lambda_{d}\right)+{\omega \lambda }_{d}S-C_{1}-y\left(\xi \text{C}-C_{1}\right)\right],\\ F_{2}\left(x,y\right)=\frac{\text{d}y}{\text{d}t}=y\left(1-y\right)\left[x\left(\Pi_{R}^{YY}-\Pi_{R}^{YN}\right)+\left(1-x\right)\left(\Pi_{R}^{NY}-\Pi_{R}^{NN}\right)\right],\\ F_{2}\left(x,y\right)=y\left(1-y\right)\left[S\left(P_{r}-\omega \right)\left(1-\lambda_{r}\right)-C_{1}+C_{1}x-\text{C}x\left(1-\xi \right)\right]. \end{array}$$

In the above, the evolution equilibrium points (0, 0), (0, 1), (1, 0), (1, 1), and (*x*_0_, *y*_0_) of the system are obtained by d*x*/d*t*=0, d*y*/d*t*=0.

(15) $$\begin{array}{c} x_{0}=\frac{S\left(P_{r}-\omega \right)\left(1-\lambda_{r}\right)-C_{1}}{\left(1-\xi \right)C-C_{1}},\\ y_{0}=\frac{P_{d}S\left(1-\lambda_{d}\right)+{\omega \lambda }_{d}S-C_{1}}{\xi \text{C}-C_{1}}. \end{array}$$

The Jacobian matrix of the system is expressed in formula (4).

(16) $$\begin{array}{c} de\;tJ=\left[\begin{array}{cc} \frac{\partial F_{1}\left(x,y\right)}{\partial x} & \frac{\partial F_{1}\left(x,y\right)}{\partial y}\\ \frac{\partial F_{2}\left(x,y\right)}{\partial x} & \frac{\partial F_{2}\left(x,y\right)}{\partial y} \end{array}\right]=\left[\begin{array}{cc} D_{11} & D_{12}\\ D_{21} & D_{22} \end{array}\right]=D_{11}D_{22}-D_{12}D_{21}>0,\\ D_{11}=\left(1-2x\right)\left[P_{d}S\left(1-\lambda_{d}\right)+{\omega \lambda }_{d}S-C_{1}-y\left(\xi \text{C}-C_{1}\right)\right],\\ D_{12}=x\left(1-x\right)\left(C_{1}-\xi \text{C}\right),\\ D_{21}=y\left(1-y\right)\left(C_{1}-\text{C}+\xi \text{C}\right),\\ D_{22}=\left(1-2y\right)\left[S\left(P_{r}-\omega \right)\left(1-\lambda_{r}\right)-C_{1}+C_{1}x-\text{C}x\left(1-\xi \right)\right]. \end{array}$$

The trace of the matrix is computed using the following formula:

(17) $$\begin{array}{c} trJ=D_{11}+D_{22}. \end{array}$$

According to the verification method of the evolutionary stability strategy proposed by Friedman, the local stability points are determined by analyzing the symbols of *de*  *tJ* and *trJ* on five equilibrium points. The judgment conditions are as follows:

(18) $$\begin{array}{c} \det\;J>0\text{ and }trJ=D_{11}+D_{22}<0. \end{array}$$

If the equilibrium point satisfies condition (6), it is a locally stable point (ESS). Through analysis, the equilibrium results can be obtained as shown in Table 5. As can be seen from Table 5, the final evolution results are locally stable at (0, 0) and (1, 1). The evolutionary phase is shown in Figure 3.

As shown in Figure 3, when the initial state is located in the ABEC area, the system will converge to *A* (0, 0); that is, the brand adopts the dual-channel model, while the franchisee does not provide showroom services. When the initial state is located in the CEBD area, the system will converge to *D* (1, 1); that is, the brand adopts the O2O model, while the franchisee provides showroom services.

### 5.2. Analysis on Stability of Evolutionary Equilibrium

To reflect the evolution process of service sharing intention between the brand and the franchisee, the paper analyzes the influence of the change of relevant parameters on the cooperation intention of both parties through numerical simulation. Let us assume that the service level *S* = 1, offline retail price *P*_*r*_ = 4, online direct selling price *P*_*d*_ = 3, the wholesale price *ω* = 2, the cost sharing proportion of the brand *ξ* = 0.5, offline free riding coefficient *λ*_*d*_ = 0.5, online free riding coefficient *λ*_*r*_ = 0.6, service sharing total cost *C* = 1, and the service cost *C*_1_ = 3.

**Conclusion 8 .**

Price sensitivity coefficient *β* between channels does not affect the evolutionary game. In the long run, the price difference between channels has an impact on the willingness of the brand and the franchisee to cooperate in service sharing.

It is a common and long-term phenomenon that the direct sales price *P*_*d*_ in the online channel is lower than the retail price *P*_*r*_ in the offline channel. Therefore, in the long run, the price difference between channels will not have a significant impact on the evolution of decisions of both parties.

**Conclusion 9 .**

The variation of free riding coefficient *λ*_**d**_  in offline channels has little impact on the initial intention of the brand, while the initial intention of the franchisee will decline with the decrease of free riding coefficient  *λ*_*d*_. In the long run, with the decrease of  *λ*_*d*_, the cooperative intention of service sharing between the brand and the franchisee becomes stronger and stronger. The results are shown in Figure 4.

The critical value of the free riding coefficient *λ*_*d*_ in offline channels is between 0.6 and 0.7. In case *λ*_*d*_ is less than the critical value, the brands' willingness to cooperate in service sharing continues to rise, while the cooperative intention of service sharing of the franchisee increases rapidly after an initial slight decline, and, finally, both parties tend to stabilize at (1, 1). At this point, as *λ*_*d*_ decreases, both parties converge to (1, 1). In case *λ*_*d*_ is greater than the critical value, the cooperation willingness of the franchisee service sharing continues to decline, while the cooperation willingness of brand service sharing decreases rapidly after a slight initial increase, and, finally, both parties tend to stabilize at (0, 0). At this point, with the increase of *λ*_*d*_, both parties converge to (0, 0) faster. This is because the change of free riding coefficient *λ*_*d*_  of offline channels mainly affects the revenue of the franchisees. The smaller *λ*_*d*_ is, the lower the initial willingness of the franchisee to share services is. However, as *λ*_*d*_ continuous to decrease, so does the franchisee's profit. Therefore, the franchisees actively seek cooperation with the brand to realize service sharing and increase online to offline traffic to increase their revenue. The results are shown in Figure 4.

**Conclusion 10 .**

The variation of free riding coefficient *λ*_*r*_ in online channels has little influence on the initial willingness of the franchisee. However, the initial willingness of the brand will decrease with the decrease of  *λ*_*r*_. In the long run, the free riding coefficient *λ*_*r*_ of online channels is an interval value. When  *λ*_*r*_ ∈ [0.6,  0.7], the brand and the franchisee have the strong cooperative intention of service sharing. The results are shown in Figure 5.

When *λ*_*r*_ ∈ [0.6,  0.7], the cooperative willingness of brand owners to share their services continues to rise, while the cooperative willingness of franchisees to share their services rises rapidly after an initial small decline, and eventually both sides converge to a stable point (1, 1). At this point, the smaller *λ*_*r*_ is, the faster the convergence rate is. When  *λ*_*r*_ ∉ (0.5,  0.8), the willingness of the franchisee to cooperate in service sharing continues to decline, while the willingness of the brand to cooperate in service sharing decreases after the slight initial increase; eventually both parties will reach a stable point (0, 0). This is because, with the increase of *λ*_*r*_  gradually beyond the range, although the willingness of the brand service sharing is more and more strong, the franchisees are more willing not to provide showroom services due to increasing profit loss caused by free riding in online channels. As *λ*_*r*_ decreases and gradually exceeds the interval range, the profit growth of the brand due to free riding also decreases, leading to a gradual decrease in the willingness to share services.

**Conclusion 11 .**

The change cost sharing coefficient *ξ* of the brand has little influence on the initial willingness of the brand and the franchisee. In the long run, the greater the cost sharing coefficient  *ξ* of the service sharing brand, the stronger the willingness of service sharing. The results are shown in Figure 6.

The *ξ* threshold is between 0.4 and 0.5. When *ξ* is less than the critical value, the franchisee's willingness to provide showroom services continues to decline, while the brand's willingness to cooperate in service sharing decreases rapidly after a slight initial increase, and, finally, both parties tend to (0, 0). At this point, with the decrease of *ξ* value, both parties accelerate to converge towards point (0, 0). With the decrease of *ξ* value, the convergence of both sides to (0, 0) is accelerated. When *ξ* is greater than this critical value, the cooperation willingness of service sharing of the brand continues to rise, while the cooperation willingness of service sharing of the franchisee increases rapidly after a slight initial decline, and, finally, both parties tend to stabilize at (1, 1). The speed of convergence to (1, 1) increases with the increase of *ξ*. This is due to the lower initial willingness of the franchisee to share services compared to the brand. With the increase of *ξ*, the greater the proportion of sharing cost of the brand is, the more willing franchisees are to share service.

## 6. Conclusion

Online and offline services have their characteristics, including information services such as products and prices in online channels, as well as personalized experience services in offline channels. Therefore, to improve customer consumption experience, cooperation between online and offline channels to achieve service sharing is imperative. However, the competition between brands and franchisees and the bidirectional free riding phenomenon between channels make the problem of service sharing between channels more complicated. In this paper, the cooperative intention of service sharing between channels is taken as the starting point, and the static Stackelberg game and dynamic evolutionary game double-equilibrium linkage model is constructed, and the influence factors of bidirectional free riding degree, price sensitivity between channels, and service sharing cost sharing ratio are introduced. Firstly, this paper analyzes the short-term optimal strategy and equilibrium strategy of the brand and the franchisee based on static equilibrium results and concludes that the prisoner's dilemma will lead to a loss-loss result and the Pareto optimality will lead to a win-win result. Secondly, the dynamic evolutionary game is derived from the long-term stable strategies of brand owners and franchisees. Finally, the study analyzes the effects of relevant parameter changes on static and dynamic equilibrium outcomes. This study has some reference value for supplier members to implement interchannel service sharing operation management. At the same time, the model proposed in this paper is easy to implement, the implementation cost is low, and the computational complexity belongs to the class P problem, which is a practical problem that can be solved on the computer. The future research direction of interchannel service sharing under the situation of power structure is dominated by offline physical stores, random demand, and service level changing with the service cost.

## Figures and Tables

**Figure 1:** Dual-channel supply chain service sharing decision chart.

**Figure 2:** System equilibrium strategy under different cost combination.

**Figure 3:** Evolutionary phase.

**Figure 4:** The influence of *λ*_*d*_  variation on evolution results.

**Figure 5:** The influence of *λ*_*r*_  variation on evolution results.

**Figure 6:** The influence of *ξ*  variation on evolution results.

**Table 1:** Notations for the models.

Notation	Description
*ω*	Wholesale price
*P*_*r*_	Retail price in the offline channel
*P*_*d*_	Direct selling price in the online channel
*S*_*d*_	The brand provides drainage services
*S*_*r*_	The franchisee provides showroom services
*λ*_*d*_(*λ*_*r*_)	The free riding coefficient in the offline (online) channel
*β*	The price sensitivity coefficient between channels
*ξ*	The cost sharing ratio of the brand
*C*_1_	Single-channel service cost
*C*	Dual-channel service sharing costs
*Q*_*d*_(*Q*_*r*_)	The demands of online (offline) channels
Π_*M*_(Π_*R*_)	The profits of the brand (the franchisee)

**Table 2:** Optimal pricing under each strategy combination.

Strategy	*ω* ^*∗*^	*P*_*d*_^*∗*^	*P*_*r*_^*∗*^
*G* ^*N*^ *H* ^*N*^	1/2(1 − *β*)	1/2(1 − *β*)	(3 − *β*)/4(1 − *β*)
*G* ^*N*^ *H* ^*Y*^	1/2(1 − *β*) − *Sλ*_*r*_/2(1+*β*)+*S*/2(1 − *β*^2^)	1/2(1 − *β*)+*Sλ*_*r*_/2(1+*β*)+*Sβ*/2(1 − *β*^2^)	(3 − *β*)/4(1 − *β*) − *Sλ*_*r*_(3+*β*)/4(1+*β*)+*S*(3 − *β*^2^)/4(1 − *β*^2^)
*G* ^*Y*^ *H* ^*N*^	1/2(1 − *β*)+*Sλ*_*d*_/2(1+*β*)+*Sβ*/2(1 − *β*^2^)	1/2(1 − *β*) − *Sλ*_*d*_/2(1+*β*)+*S*/2(1 − *β*^2^)	(3 − *β*)/4(1 − *β*)+*Sλ*_*d*_(3+*β*)/4(1+*β*)+*Sβ*/2(1 − *β*^2^)
*G* ^*Y*^ *H* ^*Y*^	1/2(1 − *β*)+*S*/2(1 − *β*) − *Sλ*/2(1+*β*)	(1+*S*)/2(1 − *β*)+*Sλ*/2(1+*β*)	(1+*S*)(3 − *β*)/4(1 − *β*) − *Sλ*(3+*β*)/4(1+*β*)

In the above table, *λ*=*λ*_*r*_ − *λ*_*d*_.

**Table 3:** Optimal profit under each strategy combination.

Strategy	Π_*M*_^*∗*^	Π_*R*_^*∗*^
*G* ^*N*^ *H* ^*N*^	(3+*β*)/8(1 − *β*)	1/16
*G* ^*N*^ *H* ^*Y*^	(3+*β*)+2*S*(1+*β*)/(8(1 − *β*)) − (2*S*^2^*λ*_*r*_(1 − *β*) − *S*^2^*λ*_*r*_^2^(3 − *β*))/(8(1+*β*))+(*S*^2^+*S*^2^*β*^2^)/(8(1 − *β*^2^))+(*Sλ*_*r*_)/4	(1+*S* − *Sλ*_*r*_)^2^/16 − *C*_1_
*G* ^*Y*^ *H* ^*N*^	(2*S*^2^)/(8(1 − *β*^2^))+(3+*β*+4*S*)/(8(1 − *β*)) − (4*S*^2^*λ*_*d*_ − *S*^2^*λ*_*d*_^2^(3 − *β*))/(8(1+*β*)) − (*Sλ*_*d*_)/4 − *C*_1_	(1+*Sλ*_*d*_)^2^/16
*G* ^*Y*^ *H* ^*Y*^	(1+*S*)^2^(3+*β*)/8(1 − *β*)+*S*^2^*λ*^2^(3 − *β*)/8(1+*β*)+*Sλ*(1+*S*)/4 − *ξC*	(1+*S* − *Sλ*)^2^/16 − (1 − *ξ*)*C*

In the above table, *λ*=*λ*_*r*_ − *λ*_*d*_.

**Table 4:** Payoff matrix of the brand and the franchisee.

The brand	The franchisee	
	Showroom service (*y*)	No showroom service (1 − *y*)
O2O model (*x*)	(Π_*M*_^*YY∗*^, Π_*R*_^*YY∗*^)	(Π_*M*_^*YN∗*^, Π_*R*_^*YN∗*^)
Dual-channel model(1 − *x*)	(Π_*M*_^*NY∗*^, Π_*R*_^*NY∗*^)	(Π_*M*_^*NN∗*^, Π_*R*_^*NN∗*^)

**Table 5:** Equilibrium point local stability.

Equilibrium point	det*J*	*trJ*	Stability
(0, 0)	+	−	ESS
(0, 1)	+	+	Unstable
(1, 0)	+	+	Unstable
(1, 1)	+	−	ESS
(*x*_0_, *y*_0_)	−	0	Saddle point

## Data Availability

The data used to support the findings of this study are available from the corresponding author upon request.

## Appendix

### A. The Process of Proving Propositions

Proof of Propositions 1 and 2: This paper assumes that the brand is the Stackelberg leader of the supply chain and the franchisee is the follower. The optimal pricing and profit of the four decision-making combinations (*G*^*N*^*H*^*N*^, *G*^*N*^*H*^*Y*^, *G*^*Y*^*H*^*N*^, and *G*^*Y*^*H*^*Y*^) are obtained by reverse induction. Profits of the brand and the franchisee in strategy *G*^*N*^*H*^*N*^ are shown in the two following equations:

(A.1) $$\begin{array}{c} \Pi_{M}=P_{d}\left(1-P_{d}+\beta P_{r}\right)+\omega \left(1-P_{r}+\beta P_{d}\right). \end{array}$$

(A.2) $$\begin{array}{c} \Pi_{R}=\left(P_{r}-\omega \right)\left(1-P_{r}+\beta P_{d}\right). \end{array}$$

The brand, as Stackelberg's leader, first determines the wholesale price *ω*  and the online direct selling price  *P*_*d*_. Then, the offline franchisee, as a follower, sets its retail price *P*_*r*_ according to the decisions of the brand. The authors solved this problem by backward induction. The franchisees make the first decisions. The authors can produce the result that d^2^Π_*R*_/d*P*_*r*_^2^=−2 < 0 according to equation (A.2). Therefore, Π_*R*_ is a strictly concave function of  *P*_*r*_, and there exists a unique optimal retail price *P*_*r*_=1/2(1+*ω*+*βP*_*d*_) about *ω* and  *P*_*d*_. Then, by substituting it into (A.1), the authors can obtain the following profit function of the brand:

(A.3) $$\begin{array}{c} \Pi_{M}=\frac{1}{2}\left(\omega -\omega^{2}+2P_{d}+\beta P_{d}+2\beta \omega P_{d}-2P_{d}^{2}+\beta^{2}P_{d}^{2}\right). \end{array}$$

The Hessian matrix for *ω*,  *P*_*d*_ profit function Π_*M*_ for the brand is as follows:

(A.4) $$\begin{array}{c} H=\left[\begin{array}{cc} \frac{\partial^{2}\Pi_{M}}{\partial \omega^{2}} & \frac{\partial^{2}\Pi_{M}}{\partial \omega \;\partial P_{d}}\\ \frac{\partial^{2}\Pi_{M}}{\partial P_{d}\partial \omega } & \frac{\partial^{2}\Pi_{M}}{\partial P_{d}{}^{2}} \end{array}\right]=\left[\begin{array}{cc} -1 & \beta \\ \beta & \frac{\left(-4+2\beta^{2}\right)}{2} \end{array}\right]. \end{array}$$

0 < *β* < 1 and *De*  *t*|*H*|=2 − 2*β*^2^ > 0. That means the Hessian matrix is negative definite. Therefore, Π_*M*_ is a strictly concave function of *ω* and *P*_*d*_, and there exists a unique optimal solution set. Make the first derivative of Π_*M*_ concerning *ω* and *P*_*d*_  equal to 0. The optimal wholesale price *ω* and direct selling price *P*_*d*_ can be obtained as follows:

(A.5) $$\begin{array}{c} \omega^{*}=\frac{1}{2\left(1-\beta \right)},\;P_{d}^{*}=\frac{1}{2\left(1-\beta \right)}. \end{array}$$

Accordingly, the authors can obtain *P*_*r*_, Π_*M*_^*∗*^, and Π_*R*_^*∗*^ as follows:

(A.6) $$\begin{array}{c} P_{r}=\frac{3-\beta }{4\left(1-\beta \right)},\Pi_{M}^{*}=\frac{3+\beta }{8\left(1-\beta \right)},\Pi_{R}^{*}\frac{1}{16}. \end{array}$$

The proof of optimal price and profit for other strategies is similar to strategy G^N^H^N^. 

### B. The Process of Proving Conclusions

Proof
of Conclusion 1. Compare the value of *ω*^*∗*^, *P*_*d*_^*∗*^ and *P*_*r*_^*∗*^ under different strategy combinations. *ω*^(*NN∗*)^=1/2(1 − *β*)、*ω*^(*NY∗*)^=1/2(1 − *β*) − *Sλ*_*r*_/2(1+*β*)+*S*/2(1 − *β*^2^).*ω*^*YN∗*^=1/2(1 − *β*)+*Sλ*_*d*_/2(1+*β*)+*Sβ*/2(1 − *β*^2^). *ω*^*YY∗*^=1/2(1 − *β*)+*S*/2(1 − *β*) − *Sλ*/2(1+*β*) . Comparing the values in pairs under the parameter scope that  0 < *β* < 1,  0 < *λ*_*d*_ < 1,0 < *λ*_*r*_ < 1 and *S* > 0, the following conclusions are drawn. When 1/2 < 1 − *λ*_*d*_ < *λ*_*r*_ < 1, thus due to *ω*^*YY∗*^ > *ω*^*YN∗*^ > *ω*^*NY∗*^ > *ω*^*NN∗*^. When 1/2 < *λ*_*r*_ < 1 − *λ*_*d*_ < 1, thus due to *ω*^*YY∗*^ > *ω*^*NY∗*^ > *ω*^*YN∗*^ > *ω*^*NN∗*^. Similarly, the following conclusion can be drawn by comparing *P*_*d*_^*∗*^ and *P*_*r*_^*∗*^. When, 1/2 < 1 − *λ*_*d*_ < *λ*_*r*_ < 1, thus due to *P*_*d*_^*YY∗*^ > *P*_*d*_^*NY∗*^ > *P*_*d*_^*YN∗*^ > *P*_*d*_^*NN∗*^, and *P*_*r*_^*YY∗*^ > *P*_*r*_^*YN∗*^ > *P*_*r*_^*NY∗*^ > *P*_*r*_^*NN∗*^. When 1/2 < *λ*_*r*_ < 1 − *λ*_*d*_ < 1, thus due to *P*_*d*_^*YY∗*^ > *P*_*d*_^*YN∗*^ > *P*_*d*_^*NY∗*^ > *P*_*d*_^*NN∗*^, and *P*_*r*_^*YY∗*^ > *P*_*r*_^*NY∗*^ > *P*_*r*_^*YN∗*^ > *P*_*r*_^*NN∗*^

Proof
of Conclusion 2. Within the parameter range, consider (1 − *ξ*)*C* < *C*_1_  and  *C* < *C*_1_. By comparing the optimal profit of different strategy combinations, the optimal strategy of the brand and the franchisee is obtained. Due to Π*M*^*NN∗*^=(3+*β*)/8(1 − *β*), Π*M*^*NY∗*^=(3+*β*+2*S*(1+*β*))/8(1 − *β*) − 2*S*^2^*λ*_*r*_(1 − *β*) − *S*^2^*λ*_*r*_^2^(3 − *β*)/8(1+*β*)+*S*^2^+*S*^2^*β*^2^/8(1 − *β*^2^)+*Sλ*_*r*_/4, Π_*M*_^*YN∗*^=(2*S*^2^)/8(1 − *β*^2^)+3+*β*+4*S*/8(1 − *β*) − 4*S*^2^*λ*_*d*_ − *S*^2^*λ*_*d*_^2^(3 − *β*)/8(1+*β*) − (*Sλ*_*d*_)/4 − *C*_1_, Π_*M*_^*YY∗*^=(1+*S*)^2^(3+*β*)/8(1 − *β*)+*S*^2^*λ*^2^(3 − *β*))/8(1+*β*)+*Sλ*(1+*S*)/4 − *ξC*, and *λ*=*λ*_*r*_ − *λ*_*d*_, Π_*M*_^*NN∗*^ < Π_*M*_^*NY∗*^ and Π_*M*_^*YN∗*^ <  Π_*M*_^*YY∗*^ are permanently established. Then, by comparing Π_*M*_^*NY∗*^ and Π_*M*_^*YY∗*^, the authors can get the following: when *C* < *E*_1_,  Π_*M*_^*NY∗*^ < Π_*M*_^*YY∗*^; and when >*E*_1_,  Π_*M*_^*NY∗*^ > Π_*M*_^*YY∗*^ . This shows that, for the brand, when *C* < E_1_, Π_*M*_^*YY∗*^ is the largest among the four strategies. At this time, *G*^*Y*^*H*^*Y*^ is the optimal strategy. When  *C* > E_1_, Π_*M*_^*NY∗*^ is the largest among the four strategies. At this time, *G*^*N*^*H*^*Y*^ is the optimal strategy. Similarly, Π_*R*_^*NN∗*^ < Π_*R*_^*YN∗*^ and Π_*R*_^*NY∗*^ < Π_*R*_^*YY∗*^ are permanently established. Then, by comparing Π_*R*_^*YN∗*^ and Π_*R*_^*YY∗*^, when *C* < *E*_2_,  Π_*R*_^*YN∗*^ < Π_*R*_^*YY∗*^; and when *C* > *E*_2_,  Π_*R*_^*YN∗*^ > Π_*R*_^*YY∗*^. This shows that, for the brand, when  C < E_2_, Π_*R*_^*YY∗*^ is the largest among the four strategies. At this time, *G*^*Y*^*H*^*Y*^ is the optimal strategy. When  C > E_2_, Π_*R*_^*YN∗*^ is the largest among the four strategies. At this time, *G*^*Y*^*H*^*N*^ is the optimal strategy.

Proof
of Conclusion 3. Nash equilibrium is obtained by using the game profit matrix of the brand and the franchisee. For the equilibrium decision of the brand, compare Π_*M*_^*NN∗*^ with Π_*M*_^*YN∗*^ and Π_*M*_^*NY∗*^ with Π_*M*_^*YY∗*^, respectively. When *C*_1_ > *E*_3_,  Π_*M*_^*NN∗*^ > Π_*M*_^*YN∗*^; and when  C_1_ < E_3_, Π_*M*_^*NN∗*^ < Π_*M*_^*YN∗*^. When  *C* > E_1_, Π_*M*_^*NY∗*^ > Π_*M*_^*YY∗*^；and when *C* < E_1_, Π_*M*_^*NY∗*^ < Π_*M*_^*YY∗*^. Similarly, for the equilibrium decision of the franchisee, compare Π_*R*_^*NN∗*^  with Π_*R*_^*NY∗*^ and Π_*R*_^*YN∗*^ with Π_*R*_^*YY∗*^, respectively. When C_1_ > E_4_, Π_R_^NN*∗*^ > Π_R_^NY*∗*^; and when  C_1_ < E_4_, Π_R_^NN*∗*^ < Π_R_^NY*∗*^. When  *C* > E_2_,  Π_*R*_^*YN∗*^ > Π_*R*_^*YY∗*^; and when  *C* < E_2_,  Π_*R*_^*YN∗*^ < Π_*R*_^*YY∗*^. When *C* < *E*_2_ and *C*_1_ < *E*_4_, Π_*M*_^*NN*^ < Π_*M*_^*YN*^,  Π_*M*_^*NY*^ < Π_*M*_^*YY*^ and Π_*R*_^*YN*^ < Π_*R*_^*YY*^, so *G*^*Y*^*H*^*Y*^ is the unique Nash equilibrium solution to the system. Similarly, the unique Nash equilibrium solution to other (*C*, *C*_1_) combinations can be obtained. However, when *C* < *E*_2_ and  *C*_1_ > *E*_3_,  Π_*M*_^*NN*^ > Π_*M*_^*YN*^,  Π_*M*_^*NY*^ < Π_*M*_^*YY*^,  Π_*R*_^*NN*^ > Π_*R*_^*NY*^ and Π_*R*_^*YN*^ < Π_*R*_^*YY*^, there are two Nash equilibrium solutions to the system, that is, *G*^*N*^*H*^*N*^ and *G*^*Y*^*H*^*Y*^. Combined with Conclusion 2, when the cost of shared service *C* is small, both the brand and the franchisee prefer strategy *G*^*Y*^*H*^*Y*^ to achieve win-win cooperation. In this paper, *G*^*Y*^*H*^*Y*^ strategy is selected for study. When *C* < *E*_2_ and  *C*_1_ > *E*_3_,  Π_*M*_^*NN*^ < Π_*M*_^*YN*^,  Π_*M*_^*NY*^ > Π_*M*_^*YY*^,  Π_*R*_^*NN*^ < Π_*R*_^*NY*^ and Π_*R*_^*YN*^ > Π_*R*_^*YY*^, there are also two Nash equilibrium solutions to the system, that is, *G*^*N*^*H*^*Y*^ and *G*^*Y*^*H*^*N*^. Considering that, compared with franchisees, brand owners have stronger cooperative intention of service sharing, only strategy *G*^*Y*^*H*^*N*^ is studied in this paper.

Proof
of Conclusions 4 and 5.

(B.1) $$\begin{array}{c} \frac{\partial E_{1}}{\partial \lambda_{r}}=\frac{S^{2}\left(2+\left(-3+\beta \right)\lambda_{d}\right)}{4\left(1+\beta \right)\xi }>0，\;\frac{\partial E_{1}}{\partial \lambda_{d}}=-\frac{S\left(\left(1+S\right)\left(1+\beta \right)+S\left(-3+\beta \right)\lambda_{d}-S\left(-3+\beta \right)\lambda_{r}\right)}{4\left(1+\beta \right)\xi }<0,\\ \frac{\partial E_{2}}{\partial \lambda_{r}}=\frac{S\left(S\lambda_{r}-1-S-S\lambda_{d}\right)}{8\left(1-\xi \right)}<0,\;\frac{\partial E_{2}}{\partial \lambda_{d}}=\frac{S^{2}\left(1-\lambda_{r}\right)}{8\left(1-\xi \right)}>0,\\ \frac{\partial E_{3}}{\partial \lambda_{d}}=-\frac{S\left(1+2S+\beta -S\left(3-\beta \right)\lambda_{d}\right)}{4\left(1+\beta \right)}<0,\;\frac{\partial E_{4}}{\partial \lambda_{r}}=\frac{1}{8}S\left(S\lambda_{r}-1-S\right)<0. \end{array}$$

It can be seen that when *λ*_*d*_ decreases, *E*_1_ and *E*_3_ increase, and *E*_2_  decreases, the system equilibrium strategy tends to be strategy *G*^*Y*^*H*^*N*^. When *λ*_*d*_ increases, *E*_1_ and *E*_3_ decrease, and *E*_2_ increases, the system equilibrium strategy tends to be strategy *G*^*Y*^*H*^*Y*^. Similarly, when *λ*_*r*_ decreases, *E*_2_ and *E*_4_ increase, and *E*_1_ decreases, the system equilibrium strategy tends to be strategy *G*^*Y*^*H*^*Y*^. When *λ*_*r*_ increases, *E*_2_ and *E*_4_ decrease, and *E*_1_ increases, the system equilibrium strategy tends to be strategy *G*^*Y*^*H*^*N*^. The proof of Conclusions 6 and 7 is similar to that of Conclusion 4.
